# Modeling Cancer Remission Time Data by Means of the Max Erlang Binomial Distribution

**DOI:** 10.1155/2021/9932729

**Published:** 2021-09-24

**Authors:** Bogdan Gheorghe Munteanu

**Affiliations:** Department of Fundamental Sciences, Henri Coandă Air Force Academy, Brașov, Romania

## Abstract

In this paper, a statistical simulation algorithm for the power series distribution, called the Max Erlang Binomial distribution, is proposed, analyzed, and tested for bladder cancer remission time data. In order to present the simulation technique, the EM algorithm for statistical estimation aimed at estimating the model parameters is described.

## 1. Introduction

The introduction of this new (generalized) distribution addresses reliability problems when lifetime can be expressed as the maximum or minimum of a sequence of independent and identically distributed (iid) random variables, which represents the system components' risk times. In recent years, some researchers have proposed a series of new distributions for the maximum and minimum of a sequence of iid random variables. For example, Adamidis and Loukas [1], Kus [2], Tahmasbi and Rezaei [3], Louzada et al. [4], and Cancho et al. [5] were interested in determining the maximum or minimum distribution when the components in a sequence of iid random variables are exponentially distributed, and a number of components are of a discrete type. Next, Flores et al. [6] treated the distribution of a vector's maximum with components that are exponentially distributed in a random number of a power series distribution type. This type of distribution is called the complementary exponential power series (CEPS) distribution. Also, Morais and Barreto-Souza [7] considered analyzing the Weibull distribution class by means of the power series distribution class (WPS). Recently, Louzada et al. [8] have developed a mathematical model that unifies the procedure for obtaining a distribution of the maximum and minimum of a sequence of iid random variables of the absolutely continuous type in a random number *N* characterized by the generating function. But the problem of determining the general formula when the random variable *N* forms a part of a power series distributions remains unsolved.

In this paper, the simulation algorithms for these family distributions are proposed. This study is intended as a completion of the research by Balkema and de Haan (1974), Bryson (1974), Ahsanullah (1991), Balakrishnan and Ahsanullah (1994), Childs and others (2001), Al Awadhi and Ghitany (2001, 2007), Zahrani and Harbi (2013), Al-Zahrani and Sagor (2014), Tahir and Cordeiro ([9], 2016), Hassan and Abd-Elfattah (2016), and Munteanu ([10], 2013). The above-mentioned algorithm was implemented by means of the Eclipse SDK programming environment.

This work has the following structure: Section 2 defines the mathematical properties of the Max Erlang Binomial power series distribution (the cumulative distribution function, the probability density function, the mean, and variance). The simulation techniques targeting the Max Erlang Binomial distribution are analyzed and formulated in Section 3, with results validation via the Pearson test. In Section 4, the simulation algorithm for the Max Erlang Binomial distribution parameters is proposed and tested using the method of the maximum likelihood estimation.  Section 5 discusses an application of the proposed distribution using a real-life dataset. Lastly, in Section 6, some useful conclusions are drawn.

## 2. Development of the Mathematical Model

In [11], the properties of a new power distribution type series, called the Max Erlang Binomial (MaxErlB), are introduced and researched. As a mathematical model, this distribution describes the probabilistic behavior of lifetimes, widely used in researching the reliability of systems. In [11], this distribution is presented as the distribution of the maximum value in a random volume sample *Z* from a statistical population, Erlang distributed, where *Z* is a binomially distributed, zero-truncated random variable. Formally, things are presented as follows.

Let us consider the random variable *Z* such that *ℙ*(*Z* ∈ {1, 2, ⋯}) = 1.

**Definition 1 ([12]).**

We say that the random variable *Z* has a power series distribution if

(1) $$\begin{array}{c} \mathbb{P}\left(Z=z\right)=\frac{a_{z}\Theta^{z}}{A\left(\Theta \right)},z=1,2,\cdots ;\Theta \in \left(0,\tau \right), \end{array}$$

where *a*_1_, *a*_2_, ⋯ are nonnegative real numbers, *τ* is a positive number bounded by the convergence radius of power series (series function) *A*(Θ) = ∑_*z*≥1_ *a*_*z*_Θ^*z*^, ∀Θ ∈ (0, *τ*), and Θ is the *power parameter* of the distribution (Table 1).

PSD denotes the power series distribution function families. If the random variable *Z* has the distribution in Equation (1), then we write *Z* ∈ PSD.

We consider that *X*_*i*_ ~ Erlang(*k*, *λ*), *k* ∈ *ℕ*, *k* ≥ 1, *λ* > 0, where (*X*_*i*_)_*i*≥1_ are iid random variables with the distribution function *F*_*X*_*i*__(*x*) ≡ *F*_*Erl*_(*x*) = 1 − ∑_*i*=0_^*k*−1^ ((*λx*)^*i*^/*i*!)*e*^−*λx*^, *x* > 0, and the probability density function *f*_*X*_*i*__(*x*) ≡ *f*_Erl_(*x*) = (*λ*^*k*^*x*^*k*−1^*e*^−*λx*^/(*k* − 1)!), *x* > 0.

We note that *U*_Erl_ = max {*X*_1_, *X*_2_, ⋯, *X*_*Z*_}.

The results in this section are obtained using the general framework in [13], for which reason some proofs are not presented.

**Proposition 1 (see [11]).**

If the random variable *U*_Erl_ = max{*X*_1_, *X*_2_, ⋯, *X*_*Z*_}, where (*X*_*i*_)_*i*≥1_ are nonnegative iid random variables, *X*_*i*_ ~ Erlang(*k*, *λ*), *k* ∈ *ℕ*, *k* ≥ 1, *λ* > 0 and *Z* ~ Binom^∗^(*n*, *p*), *Z* ∈ *PSD*, *n* ∈ {1, 2⋯}, with *A*(Θ) = (Θ + 1)^*n*^ − 1, Θ = (*p*/(1 − *p*)), *p* ∈ (0, 1), Θ ∈ (0, *τ*), *τ* > 0, the random variables (*X*_*i*_)_*i*≥1_ and Z being independent; then, the cumulative distribution functions and the probability density function of the random variable *U*_ErlB_ are the following:

(2) $$\begin{array}{c} U_{\text{ErlB}}\left(x\right)=\frac{{\left(1-pe^{-\lambda x}\sum_{i=0}^{k-1}\;\left({\left(\lambda x\right)}^{i}/i!\right)\right)}^{n}-{\left(1-p\right)}^{n}}{1-{\left(1-p\right)}^{n}},x>0, \end{array}$$

(3) $$\begin{array}{c} u_{\text{ErlB}}\left(x\right)=\frac{np\lambda^{k}x^{k-1}e^{-\lambda x}{\left(1-pe^{-\lambda x}\sum_{i=0}^{k-1}\;\left({\left(\lambda x\right)}^{i}/i!\right)\right)}^{n-1}}{1-{\left(1-p\right)}^{n}},x>0. \end{array}$$

**Definition 2 (see [11]).**

We say that the random variable *U*_ErlB_ has a Max Erlang Binomial power series distribution with parameters *k*, *λ*, *n*, and *p* (*U*_ErlB_ ~ MaxErlB (*k*, *λ*, *n*, *p*)), if it has the cumulative distribution function (cdf) defined by Equation (2) and probability density function (pdf) defined by Equation (3).

The numerical characteristics (mean, variance) of a random variable with a MaxErlB distribution, in a particular case (*k* = 2), are presented in the following result:

**Proposition 2 .**

The mean and variance of the random variable *U*_ErlB_ ~ MaxErlB(2, *λ*, *n*, *p*), *λ* > 0, *n* ∈ {1, 2⋯}, *p* ∈ (0, 1), are characterized by the following relations:

(4) $$\begin{array}{c} EU_{\text{ErlB}}=\frac{n}{\lambda \left[1-{\left(1-p\right)}^{n}\right]}\overset{n}{\underset{z=1}{\sum }}\;{\left(-1\right)}^{z-1}\left(\begin{array}{c} n\\ z-1 \end{array}\right)\frac{\left(z+1\right)!p^{z}}{z^{z+2}}, \end{array}$$

(5) $$\begin{array}{c} VarU_{\text{ErlB}}=\frac{n}{\lambda^{2}\left[1-{\left(1-p\right)}^{n}\right]}\left[\overset{n}{\underset{z=1}{\sum }}\;{\left(-1\right)}^{z-1}\left(\begin{array}{c} n\\ z-1 \end{array}\right)\frac{\left(z+2\right)!p^{z}}{z^{z+3}}-\frac{n}{1-{\left(1-p\right)}^{n}}{\left(\overset{n}{\underset{z=1}{\sum }}\;{\left(-1\right)}^{z-1}\left(\begin{array}{c} n\\ z-1 \end{array}\right)\frac{\left(z+1\right)!p^{z}}{z^{z+2}}\right)}^{2}\right]. \end{array}$$

**Proof**

After Equation (3) and the definition of the mean, we obtain

(6) $$\begin{array}{c} EU_{\text{ErlB}}=\frac{np\lambda^{2}}{1-{\left(1-p\right)}^{n}}\int_{0}^{\infty }\;x^{2}e^{-\lambda x}{\left(1-pe^{-\lambda x}\left(1+\lambda x\right)\right)}^{n-1}dx, \end{array}$$

where ${\left(1-pe^{-\lambda x}\left(1+\lambda x\right)\right)}^{n-1}=\sum_{z=1}^{n}\;{\left(-1\right)}^{z-1}\left(\begin{array}{c} n\\ z-1 \end{array}\right)p^{z-1}{\left(1+\lambda x\right)}^{z-1}e^{-\left(z-1\right)\lambda x}$, as developed by Newton's binomial. A sum of *n*-integrals then can be solved with elementary methods (method of integration by parts), which leads to Equation (4).

Similarly, evaluating the second-order moment

(7) $$\begin{array}{c} EU_{\text{ErlB}}^{2}=\frac{np\lambda^{2}}{1-{\left(1-p\right)}^{n}}\int_{0}^{\infty }\;x^{3}e^{-\lambda x}{\left(1-pe^{-\lambda x}\left(1+\lambda x\right)\right)}^{n-1}dx, \end{array}$$

together with the definition of variance, leads us to Equation (5).

**Remark 1 .**

We notice that for *k* = 1, we obtain the complementary exponential distribution introduced by Flores et al. [6].

## 3. Statistical Simulation for the MaxErlB Distribution

Taking advantage of the fact that the random variable *U*_ErlB_ ~ MaxErlB(*k*, *λ*, *n*, *p*), *λ* > 0, *k*, *n* ∈ {1, 2⋯}, *p* ∈ (0, 1), has the same distribution as the random variable max_1≤*i*≤*Z*_*X*_*i*_, where (*X*_*i*_)_*i*≥1_ are iid random variables, *X*_*i*_ ~ Erlang(*k*, *λ*), *k* ∈ *ℕ*, *k* ≥ 1, *λ* > 0, and the value of the random variable *Z* ~ Binom^∗^(*n*, *p*), *p* ∈ (0, 1), *n* ∈ {1, 2, ⋯}, coincide with the value of the random variable zero-truncated binomial distributed with the same parameters, but provided this is a nonzero value, we can briefly describe the following algorithm.

### 3.1. Statistical Simulation Algorithm for the MaxErlB Distribution

**Step 1 .**

We generate a value *z*^⋆^ of the random variable *Z*^⋆^ ~ Binom(*n*, *p*), *p* ∈ (0, 1), *n* ∈ {1, 2, ⋯}

**Step 2 .**

If *z*^⋆^ = 0, then GO TO Step 1; otherwise, *z* = *z*^∗^

**Step 3 .**

For the value *z* of the random variable *Z* (generated in Steps 1 and 2), simulate the values *x*_*i*_, *i* = 1, 2, ⋯ as a values of *z*-iid random variables with distribution Erlang(*k*, *λ*), *k* ∈ *ℕ*, *k* ≥ 1, *λ* > 0

**Step 4 .**

It is considered *u*_ErlB_ = max_1≤*i*≤*z*_*x*_*i*_, STOP.

Following the simulation, we can apply the Chi-square test of concordance. Based on a test, based on the results (*u*_ErlB_^1^, *u*_ErlB_^2^, ⋯, *u*_ErlB_^*m*^), the Chi-square criterion (Pearson's criterion) is applied, and the basic and alternative hypotheses are verified, respectively:

*H*_0_: sample values (*u*_ErlB_^1^, *u*_ErlB_^2^, ⋯, *u*_ErlB_^*m*^) are values of the random variable distributed MaxErlB(2, *λ*, *n*, *p*)

*H*_1_: sample values (*u*_ErlB_^1^, *u*_ErlB_^2^, ⋯, *u*_ErlB_^*m*^) are not the values of the random variable distributed MaxErlB(2, *λ*, *n*, *p*).

The test is considered valid if the empirical value of *χ*_*c*_^2^ is less than the upper critical value of the Chi-square with (*r* − 1) − *L* = (12 − 1) − 4 = 7 freedom degrees (*χ*_0.05;7_^2^ = 14.067). The statistics of Pearson's test is calculated using the following relation:

(8) $$\begin{array}{c} \chi_{c}^{2}=\overset{r}{\underset{j=1}{\sum }}\;\frac{{\left(n_{j}-n_{0}p_{j}\right)}^{2}}{n_{0}p_{j}}, \end{array}$$

where $n_{j},j=\overset{¯}{1,r}$ represents the number of observed values in the interval [*t*_*j*−1_, *t*_*j*_), *n*_0_ = ∑_*j*=1_^*r*^ *n*_*j*_.

The probabilities *p*_*j*_ that the random variable *U*_ErlB_ takes the values in the interval [*t*_*j*−1_, *t*_*j*_) are calculated using the following relation:

(9) $$\begin{array}{c} p_{j}=U_{\text{ErlB}}\left(t_{j}\right)-U_{\text{ErlB}}\left(t_{j-1}\right)\overset{\left(2\right)}{=}\frac{1}{1-{\left(1-p\right)}^{n}}\left[{\left(1-pe^{-\lambda t_{j}}\overset{k-1}{\underset{i=0}{\sum }}\;\frac{{\left(\lambda t_{j}\right)}^{i}}{i!}\right)}^{n}-{\left(1-pe^{-\lambda t_{j-1}}\overset{k-1}{\underset{i=0}{\sum }}\;\frac{{\left(\lambda t_{j-1}\right)}^{i}}{i!}\right)}^{n}\right], \end{array}$$

where $t_{j},j=\overset{¯}{0,r-1}$ represent the ends of each interval after they have been merged.

Based on the algorithm presented above, we can notice (see Table 2) that the mean and the empirical variance of the simulation results are well approximated by the mean and the theoretical variance of the random variable *U*_ErlB_ ~ MaxErlB(2,10,3, 0.2) (Proposition 2), and the Chi-square criterion validates each time the basic hypothesis according to which the simulated values are indeed governed by this distribution.

Moreover, the validation is confirmed for samples values *m* ∈ {100,1000,10000,100000,1000000,10000000}.

The histogram of the simulated data and the plot of the probability density function of the simulated distribution (Figure 1) also confirm the validity of the basic hypothesis, but visually.

## 4. EM Algorithm for the MaxErlB Distribution

The EM algorithm introduced in 1977 in the paper [14] comes to perfect the maximum likelihood method which, in the case of processing incomplete statistical data, becomes practically unusable. Next, the algorithm is implemented for the MaxErlB(2, *λ*, 3, *p*), *λ* > 0, *p* ∈ (0, 1) distribution.

We consider the values of a sample (*x*_1_, *x*_2_, ⋯, *x*_*m*_) of size *m* a statistical population govorned by a MaxErlB distribution with the probability density function *u*_ErlB_(*x*, Ψ), *x* > 0, which depends on the parameter vector Ψ = (*λ*, *p*), given that the parameter *n* of the zero-truncated binomial distribution and the parameter *k* of the Erlang distribution are given. According to the definition of the maximum likelihood function and Equation (3), we have

(10) $$\begin{array}{c} L\left(x_{1},x_{2},\cdots ,x_{m};\Psi \right)=\overset{m}{\underset{j=1}{\prod }}\;\frac{3p\lambda^{2}x_{j}e^{-\lambda x_{j}}{\left(1-pe^{-\lambda x_{j}}-p\lambda x_{j}e^{-\lambda x_{j}}\right)}^{2}}{1-{\left(1-p\right)}^{3}}=\frac{{\left(3p\lambda^{2}\right)}^{m}e^{-\lambda \sum_{j=1}^{m}\;x_{j}}}{{\left(1-{\left(1-p\right)}^{3}\right)}^{m}}\overset{m}{\underset{j=1}{\prod }}\;x_{j}{\left(1-pe^{-\lambda x_{j}}-p\lambda x_{j}e^{-\lambda x_{j}}\right)}^{2}. \end{array}$$

To obtain the maximum likelihood equations for the MaxErlB distribution regarding the estimation $\hat{\lambda },\hat{p}$ for the parameters *λ*, *p*, we consider

(11) $$\begin{array}{c} \ln L\left(x_{1},x_{2},\cdots ,x_{m};\lambda ,p\right)=m\left(\ln3+\ln p+2\ln\lambda \right)-\lambda \overset{k-1}{\underset{i=0}{\sum }}\;x_{j}-m\ln\left(1-{\left(1-p\right)}^{3}\right)+\overset{m}{\underset{j=1}{\sum }}\;\left[\ln x_{j}+2\left(1-pe^{-\lambda x_{j}}-p\lambda x_{j}e^{-\lambda x_{j}}\right)\right]. \end{array}$$

The parameters *n* and *k* being considered known, then the equations of the method for the maximum likelihood estimation function (MLE) are characterized by the nonlinear system *S*(Ψ) = 0, where *S*(Ψ) = ((*∂*ln*L*/*∂λ*), (*∂*ln*L*/*∂p*)). Developing the system of equations *S*(Ψ) = 0, we notice that it becomes difficult to solve in relation to the unknowns *λ* and *p*. We are thus in the situation in which the application of the EM algorithm explained and analyzed by Dempster et al. [14], then expanded by McLachlan and Krishnan [15] is required. In this algorithm, the random variable *Z* is considered a random variable latency, that is, the random variable which cannot be observed directly.

For this, we consider, formally, the following sample:

(12) $$\begin{array}{c} \left(\left(x_{1},z_{1}\right),\left(x_{2},z_{2}\right),\cdots ,\left(x_{m},z_{m}\right)\right), \end{array}$$

by *m* observations of the random variable (*U*_ErlB_, *Z*).

This shows that ((*x*_1_, *z*_1_), (*x*_2_, *z*_2_), ⋯, (*x*_*m*_, *z*_*m*_)) can be interpreted as a complete set of statistics, being, in this case, a sample of incomplete data. The description of the EM algorithm supposes a known conditional mean *𝔼*(*Z*|*U*_ErlB_; Ψ), where Ψ = (*λ*, *p*).

The probability density function *u*_ErlB_(*x*, Ψ), *x* > 0, of the random variable *U*_ErlB_ wich corresponds to a complete set of data, is defined by the following relation according to the definition of probability density in the case of the maximum (see [13], Consequence 2.2):

(13) $$\begin{array}{c} u_{\text{ErlB}}\left(x\right)=\frac{\Theta \lambda^{2}xe^{-\lambda x}\left\{A^{\prime }\left[\Theta \left(1-e^{-\lambda x}-\lambda xe^{-\lambda x}\right)\right]\right\}}{A\left(\Theta \right)},x>0, \end{array}$$

In these conditions, the probability density function *u*_ErlB_(*x*, *z*) of the random variable (*U*_ErlB_, *Z*) which corresponds to a complete set of data is given by

(14) $$\begin{array}{c} u_{ErlB}\left(x,z;\Psi \right)=zf_{Erl}\left(x\right){\left(F_{Erl}\left(x\right)\right)}^{z-1}\mathbb{P}\left(Z=z\right)=\frac{za_{z}\Theta^{z}\lambda^{2}xe^{-\lambda x}{\left(1-e^{-\lambda x}-\lambda xe^{-\lambda x}\right)}^{z-1}}{A\left(\Theta \right)}, \end{array}$$

where *A*(Θ) = (1 + Θ)^*n*^ − 1, Θ = *p*/1 − *p*, *p* ∈ (0, 1), $a_{z}=\left(\begin{array}{c} n\\ z \end{array}\right)$, *z* ≤ *n*, *f*_Erl_(*x*), and *F*_Erl_(*x*), *x* > 0 are the probability density function, respectively, the cumulative distribution function which has the Erlang(*k*, *λ*), *k* ∈ *ℕ*, *k* ≥ 1, *λ* > 0 distribution.

Then, the probability density function of the random variable *Z* conditioned by the random variable *U*_ErlB_ has the following expression:

(15) $$\begin{array}{c} u_{\text{ErlB}}\left(z\left|x\right.\right)=\frac{u_{\text{ErlB}}\left(x,z\right)}{u_{\text{ErlB}}\left(x\right)}=\frac{za_{z}\Theta^{z-1}{\left(1-e^{-\lambda x}-\lambda xe^{-\lambda x}\right)}^{z-1}}{A^{\prime }\left[\Theta \left(1-e^{-\lambda x}-\lambda xe^{-\lambda x}\right)\right]}. \end{array}$$

Therefore, considering the obvious relation ∑_*z*≥1_ *z*^2^*a*_*z*_Θ^*z*−2^ = *A*′′(Θ) + (1/Θ) · *A*′(Θ), the conditional mean becomes

(16) $$\begin{array}{c} E\left(Z\left|U_{\text{ErlB}}\right.;\Psi \right)=\overset{n}{\underset{z=1}{\sum }}\;z\cdot u_{\text{ErlB}}\left(z\left|x\right.;\Psi \right)=\frac{\sum_{z=1}^{n}\;z^{2}a_{z}\Theta^{z-1}{\left(1-e^{-\lambda x}-\lambda xe^{-\lambda x}\right)}^{z-1}}{A^{\prime }\left[\Theta \left(1-e^{-\lambda x}-\lambda xe^{-\lambda x}\right)\right]}=\frac{\Theta \left(1-e^{-\lambda x}-\lambda xe^{-\lambda x}\right)}{A^{\prime }\left[\Theta \left(1-e^{-\lambda x}-\lambda xe^{-\lambda x}\right)\right]}\overset{n}{\underset{z=1}{\sum }}\;z^{2}a_{z}\Theta^{z-2}{\left(1-e^{-\lambda x}-\lambda xe^{-\lambda x}\right)}^{z-2}=\frac{\Theta \left(1-e^{-\lambda x}-\lambda xe^{-\lambda x}\right)\cdot A^{\prime \prime }\left[\Theta \left(1-e^{-\lambda x}-\lambda xe^{-\lambda x}\right)\right]}{A^{\prime }\left[\Theta \left(1-e^{-\lambda x}-\lambda xe^{-\lambda x}\right)\right]}+1. \end{array}$$

Since *Z* ~ Binom^⋆^(*n*, *p*) ∈ *PSD*, *k*, *n* ∈ {1, 2, ⋯} with *A*(Θ) = (1 + Θ)^*n*^ − 1, Θ ∈ (0, +∞), Θ = *p*/1 − *p*, *p* ∈ (0, 1), we have

(17) $$\begin{array}{c} E\left(Z\left|U_{\text{ErlB}}\right.;\Psi \right)=\frac{2p\left(1-e^{-\lambda x}-\lambda xe^{-\lambda x}\right)}{1-pe^{-\lambda x}-p\lambda xe^{-\lambda x}}+1. \end{array}$$

We describe the EM algorithm for the MaxErlB(2, *λ*, 3, *p*) distribution as an iterative process of estimating the unknown parameter Ψ = (*λ*, *p*) through Ψ^(*h*)^ = (*λ*^(*h*)^, *p*^(*h*)^) calculated for a few steps *h* ≥ 1 such that the following condition is satisfied:

(18) $$\begin{array}{c} \max\left(\left|\lambda^{\left(h\right)}-\lambda^{\left(h-1\right)}\right|,\left|p^{\left(h\right)}-p^{\left(h-1\right)}\right|\right)\leq \varepsilon , \end{array}$$

or *h* = *K* be accomplished when *ε* > 0 and *K* represents the number of preset iterations.

The steps of the EM algorithm for MaxErlB distribution are the following:

**Step 5 .**

We take *λ* = *λ*^(0)^, *p* = *p*^(0)^, *λ*^(0)^ > 0, *p*^(0)^ ∈ (0, 1)

**Step 6 . (Expectation).**

To iterate *h*, *h* ≥ 1, we calculate the mean value of *z*_*j*_^(*h* − 1)^, $j=\overset{¯}{1,m}$ according to Equation (17) for *k* = 2:

(19) $$\begin{array}{c} z_{j}^{\left(h-1\right)}=\frac{2p^{\left(h-1\right)}\left(1-e^{-\lambda^{\left(h-1\right)}x_{j}}\left(1+\lambda^{\left(h-1\right)}x_{j}\right)\right)}{1-p^{\left(h-1\right)}e^{-\lambda^{\left(h-1\right)}x_{j}}\left(1+\lambda^{\left(h-1\right)}x_{j}\right)}+1 \end{array}$$

**Step 7 . (Maximization).**

Through the maximum likelihood estimation (MLE) method, we take into consideration the following sample:

(20) $$\begin{array}{c} \left(\left(x_{1},z_{1}^{\left(h-1\right)}\right),\left(x_{2},z_{2}^{\left(h-1\right)}\right),\cdots ,\left(x_{m},z_{m}^{\left(h-1\right)}\right)\right), \end{array}$$

with the maximum likelihood function:

(21) $$\begin{array}{c} L\left(x_{1},\cdots ,x_{m},z_{1}^{\left(h-1\right)},\cdots ,z_{m}^{\left(h-1\right)};\Psi^{\left(h-1\right)}\right)=\overset{m}{\underset{j=1}{\prod }}\;u_{ErlB}\left(x_{j},z_{j}^{\left(h-1\right)};\Psi^{\left(h-1\right)}\right)=\overset{m}{\underset{j=1}{\prod }}\;\left[\frac{z_{j}^{\left(h-1\right)}x_{j}\left(\begin{array}{c} 3\\ z_{j}^{\left(h-1\right)} \end{array}\right){\left(p^{\left(h-1\right)}\right)}^{z_{j}^{\left(h-1\right)}}{\left(1-p^{\left(h-1\right)}\right)}^{3-z_{j}^{\left(h-1\right)}}}{1}\cdot \right.\left.\cdot \frac{{\left(\lambda^{\left(h-1\right)}\right)}^{2}e^{-\lambda^{\left(h-1\right)}x_{j}}{\left(1-e^{-\lambda^{\left(h-1\right)}x_{j}}\left(1+\lambda^{\left(h-1\right)}x_{j}\right)\right)}^{z_{j}^{\left(h-1\right)}-1}}{1-{\left(1-p^{\left(h-1\right)}\right)}^{3}}\right].={\left[\frac{{\left(\lambda^{\left(h-1\right)}\right)}^{2}}{1-{\left(1-p^{\left(h-1\right)}\right)}^{3}}\right]}^{m}\overset{m}{\underset{j=1}{\prod }}\;\left[z_{j}^{\left(h-1\right)}x_{j}\left(\begin{array}{c} 3\\ z_{j}^{\left(h-1\right)} \end{array}\right){\left(p^{\left(h-1\right)}\right)}^{z_{j}^{\left(h-1\right)}}{\left(1-p^{\left(h-1\right)}\right)}^{3-z_{j}^{\left(h-1\right)}}\cdot \right.\left.\cdot e^{-\lambda^{\left(h-1\right)}x_{j}}{\left(1-e^{-\lambda^{\left(h-1\right)}x_{j}}\left(1+\lambda^{\left(h-1\right)}x_{j}\right)\right)}^{z_{j}^{\left(h-1\right)}-1}\right]. \end{array}$$

Thus, we can find iteration Ψ^(*h*)^ = (*λ*^(*h*)^, *p*^(*h*)^) which estimates the parameters Ψ = (*λ*, *p*)

**Step 8 .**

We examine Equation (18). If NOT, then GO TO Step 2; otherwise, Ψ≔Ψ^(*h*)^, STOP.

Given the function

(22) $$\begin{array}{c} \ln L\left(x_{1},x_{2},\cdots ,x_{m},z_{1}^{\left(h-1\right)},z_{2}^{\left(h-1\right)},\cdots ,z_{m}^{\left(h-1\right)};\Psi^{\left(h-1\right)}\right)==2m\ln\lambda^{\left(h-1\right)}-m\ln\left[1-{\left(1-p^{\left(h-1\right)}\right)}^{3}\right]+\overset{m}{\underset{j=1}{\sum }}\;\left\{\ln\left(\begin{array}{c} 3\\ z_{j}^{\left(h-1\right)} \end{array}\right)+\ln z_{j}^{\left(h-1\right)}+z_{j}^{\left(h-1\right)}\ln p^{\left(h-1\right)}+\left(3-z_{j}^{\left(h-1\right)}\right)\ln\left(1-p^{\left(h-1\right)}\right)+\right.+\left.\ln x_{j}-\lambda^{\left(h-1\right)}x_{j}+\left(z_{j}^{\left(h-1\right)}-1\right)\ln\left[1-e^{-\lambda^{\left(h-1\right)}x_{j}}\left(1+\lambda^{\left(h-1\right)}x_{j}\right)\right]\right\}, \end{array}$$

the maximum likelihood equations are characterized by the nonlinear system *S*(Ψ^(*h* − 1)^) = ((*∂*ln*L*/*∂λ*^(*h* − 1)^), (*∂*ln*L*/*∂p*^(*h* − 1)^), namely

(23) $$\begin{array}{c} S\left(\Psi^{\left(h-1\right)}\right)\text{: }\left\{\begin{array}{c} \frac{2m}{\lambda^{\left(h-1\right)}}+\overset{m}{\underset{j=1}{\sum }}\;\left(\frac{x_{j}^{2}\lambda^{\left(h-1\right)}\left(z_{j}^{\left(h-1\right)}-1\right)e^{-\lambda^{\left(h-1\right)}x_{j}}}{1-e^{-\lambda^{\left(h-1\right)}x_{j}}\left(1+\lambda^{\left(h-1\right)}x_{j}\right)}-x_{j}\right)=0\\ -\frac{3m{\left(1-p^{\left(h-1\right)}\right)}^{2}}{1-{\left(1-p^{\left(h-1\right)}\right)}^{3}}-\frac{3m}{1-p^{\left(h-1\right)}}+\frac{\sum_{j=1}^{m}\;z_{j}^{\left(h-1\right)}}{p^{\left(h-1\right)}\left(1-p^{\left(h-1\right)}\right)}=0. \end{array}\right. \end{array}$$

Table 3 shows the results obtained from the implementation of the EM algorithm (described above), in the Octave 1.5.4 GUI programming environment. We must also emphasize that for different sample sizes (*m* ∈ {100,1000,10000,100000,1000000}), we obtain very good approximations of the parameters *λ* and *p* that characterize the MaxErlB distribution, when the parameters *k* and *n* are known.

## 5. Application

We will now consider a dataset which represents the remission times (in months) of a random sample of 128 bladder cancer patients. The dataset itself has previously been used in [16–18]. It is summarized as follows: 0.08, 2.09, 3.48, 4.87, 6.94, 8.66, 13.11, 23.63, 0.20, 2.23, 3.52, 4.98, 6.97, 9.02, 13.29, 0.40, 2.26, 3.57, 5.06, 7.09, 9.22, 13.80, 25.74, 0.50, 2.46, 3.64, 5.09, 7.26, 9.47, 14.24, 25.82, 0.51, 2.54, 3.70, 5.17, 7.28, 9.74, 14.76, 26.31, 0.81, 2.62, 3.82, 5.32, 7.32, 10.06, 14.77, 32.15, 2.64, 3.88, 5.32, 7.39, 10.34, 14.83, 34.26, 0.90, 2.69, 4.18, 5.34, 7.59, 10.66, 15.96, 36.66, 1.05, 2.69, 4.23, 5.41, 7.62, 10.75, 16.62, 43.01, 1.19, 2.75, 4.26, 5.41, 7.63, 17.12, 46.12, 1.26, 2.83, 4.33, 5.49, 7.66, 11.25, 17.14, 79.05, 1.35, 2.87, 5.62, 7.87, 11.64, 17.36, 1.40, 3.02, 4.34, 5.71, 7.93, 11.79, 18.10, 1.46, 4.40, 5.85, 8.26, 11.98, 19.13, 1.76, 3.25, 4.50, 6.25, 8.37, 12.02, 2.02, 3.31, 4.51, 6.54, 8.53, 12.03, 20.28, 2.02, 3.36, 6.76, 12.07, 21.73, 2.07, 3.36, 6.93, 8.65, 12.63, and 22.69.

Figure 2 provides the histogram of relative frequencies of a sample size which characterizes the remission times of bladder cancer, where the curve represents the pdf of the random variable *U*_ErlB_ ~ MaxErlB(2,10,3, 0.2) distribution defined by Equation (3).

## 6. Conclusion

The conclusions revealed by the present research are related to the study of power series distributions type of a maximum of a sequence of iid random variables which are found in a random number.

Also, the distribution of a maximum number of iid random variables through the PSD family, characterized by the number of the random variable in the sequence, was presented in a compact, coherent approach.

For this purpose, programs for the statistical simulation of the MaxErlB power series distributions type were developed. The validity of the maximum distributions was performed using Pearson's test of consistency and is reflected in Table 2. Describing the EM algorithm implemented in the GUI Octave 1.5.4 programming environment to estimate the parameters of the MaxErlB distribution is presented in Table 3.

A real data sequence on bladder cancer remission times was used to illustrate and compare the histogram of the relative frequencies of remission times and the probability density function plot of the remission time values that are governed by the MaxErlB distribution (Figure 2).

## Figures and Tables

**Figure 1:** Histograms of relative frequencies of samples size *m* = 1000,10000,100000,1000000 and probability density function of the simulated values that are governed by the MaxErlB(2,10,3, 0.2) distribution.

**Figure 2:** A histogram and probability density function plot for remission times of bladder cancer.

**Table 1:** The representative elements of the PSD families for various truncated distributions.

Distribution	*a*_*z*_	Θ	*A*(Θ)	*τ*
Binom^∗^(*n*, *p*)	$\left(\begin{array}{c} n\\ z \end{array}\right)$	$\frac{p}{1-p}$	(1 + Θ)^*n*^ − 1	∞
Poisson^∗^(*α*)	$\frac{1}{z!}$	*α*	*e*^Θ^ − 1	∞
Log(*p*)	$\frac{1}{z}$	*p*	−ln(1 − Θ)	1
Geom^∗^(*p*)	1	1 − *p*	$\frac{\Theta }{1-\Theta }$	1
Pascal(*k*, *p*)	$\left(\begin{array}{c} z-1\\ k-1 \end{array}\right)$	1 − *p*	${\left(\frac{\Theta }{1-\Theta }\right)}^{k}$	1
Bineg^∗^(*k*, *p*)	$\left(\begin{array}{c} z+k-1\\ z \end{array}\right)$	*p*	(1 − Θ)^−*k*^ − 1	1

**Table 2:** The validation of the MaxErlB simulation results with the application of the Chi-square test.

Sample size	Mean		Variance		Chi-square
	Theoretical	Empirical	Theoretical	Empirical	
100	0.2197	0.2080	0.0202	0.0182	2.061
1000		0.2141		0.0228	6.952
10000		0.2151		0.0217	5.317
100000		0.2170		0.0216	4.833
1000000		0.2168		0.0215	7.636
10000000		0.2167		0.0214	2.901

**Table 3:** The estimate of the parameter vector Ψ = (*λ*, *p*) of MaxErlB(2, *λ*, 3, *p*) distribution by $\hat{\Psi }=\left(\hat{\lambda },\hat{p}\right)$.

Sample size	(*λ*, *p*)	$\hat{\lambda }$	$\hat{p}$	*h*
100	(1, 0.5)	1.017	0.494	134
1000		1.030	0.518	144
10000		0.999	0.496	152
100000		0.999	0.503	150
1000000		0.998	0.497	152

## Data Availability

All data are fully available without restriction.
